# Sensitive Visual Detection of AHPND Bacteria Using Loop-Mediated Isothermal Amplification Combined with DNA-Functionalized Gold Nanoparticles as Probes

This article has been retracted.

**DOI:** 10.1371/journal.pone.0151769

**Published:** 2016-03-22

**Authors:** Narong Arunrut, Jantana Kampeera, Sarawut Sirithammajak, Piyachat Sanguanrut, Porranee Proespraiwong, Rungkarn Suebsing, Wansika Kiatpathomchai

**Affiliations:** 1 Bioengineering and Sensing Technology Laboratory, BIOTEC, National Science and Technology Development Agency (NSTDA), 113 Thailand Science Park, Phahonyothin Rd., Khlong Nueng, Khlong Luang, Pathum Thani 12120, Thailand; 2 Center of Excellence for Shrimp Molecular Biology and Biotechnology (CENTEX Shrimp), Faculty of Science, Mahidol University, Rama VI road, Bangkok 10400, Thailand; 3 Aquatic Animal Health Research Center, Charoen Pokphand Foods Pulic CO., LTD. Samutsakorn 74000, Thailand; National Cheng Kung University, TAIWAN

## Abstract

Acute hepatopancreatic necrosis disease (AHPND) is a component cause of early mortality syndrome (EMS) of shrimp. In 2013, the causative agent was found to be unique isolates of *Vibrio parahaemolyticus* (VP_AHPND_) that contained a 69 kbp plasmid (pAP1) carrying binary Pir-like toxin genes *Pir*^*vp*^*A* and *Pir*^*vp*^*B*. In Thailand, AHPND was first recognized in 2012, prior to knowledge of the causative agent, and it subsequently led to a precipitous drop in shrimp production. After VP_AHPND_ was characterized, a major focus of the AHPND control strategy was to monitor broodstock shrimp and post larvae for freedom from VP_AHPND_ by nucleic acid amplification methods, most of which required use of expensive and sophisticated equipment not readily available in a shrimp farm setting. Here, we describe a simpler but equally sensitive approach for detection of VP_AHPND_ based on loop-mediated isothermal amplification (LAMP) combined with unaided visual reading of positive amplification products using a DNA-functionalized, ssDNA-labled nanogold probe (AuNP). The target for the special set of six LAMP primers used was the VP_AHPND_ *Pir*^*vp*^*A* gene. The LAMP reaction was carried out at 65°C for 45 min followed by addition of the red AuNP solution and further incubation at 65°C for 5 min, allowing any *Pir*^*vp*^*A* gene amplicons present to hybridize with the probe. Hybridization protected the AuNP against aggregation, so that the solution color remained red upon subsequent salt addition (positive test result) while unprotected AuNP aggregated and underwent a color change from red to blue and eventually precipitated (negative result). The total assay time was approximately 50 min. The detection limit (100 CFU) was comparable to that of other commonly-used methods for nested PCR detection of VP_AHPND_ and 100-times more sensitive than 1-step PCR detection methods (10^4^ CFU) that used amplicon detection by electrophoresis or spectrophotometry. There was no cross reaction with DNA templates derived from non-AHPND bacteria commonly found in shrimp ponds (including other *Vibrio* species). The new method significantly reduced the time, difficulty and cost for molecular detection of VP_AHPND_ in shrimp hatchery and farm settings.

## Introduction

Early mortality syndrome (EMS) refers to unusually high mortality in cultivated shrimp within approximately 35 days after stocking of rearing ponds. A component of EMS is acute hepatopancreatic necrosis disease (AHPND) that was first described as acute hepatopancreatic necrosis syndrome (AHPNS) in farmed pacific white shrimp (*Penaeus vannamei*) and giant or black tiger shrimp (*Peneus monodon*) from China in 2009 [1,2]. The name was changed to AHPND when the causative agent was later discovered to be unique isolates of *Vibrio parahaemolyticus* (VP_AHPND_) that carry a 69 kbp plasmid (pAP1) that contains binary Pir-like toxin genes *Pir*^*vp*^*A* and *Pir*^*vp*^*B* [3–6]. AHPND spread from China to Vietnam, Malaysia, Thailand, Mexico and the Philippines [7]. After its first appearance in Thailand on the eastern coast of the Gulf of Thailand in late 2012, shrimp production dropped from a high of approximately 600,000 metric tons in 2011 to less than 200,000 in 2014 (FishStat; Food and Agriculture Organization of the United Nations) from a combination AHPND mortality and farmer reluctance to stock ponds until a solution was found.

Recently, molecular tools such as polymerase chain reaction (PCR) based on targeting the toxin genes *Pir*^*vp*^*A* and *Pir*^*vp*^*B* have been reported for early detection and prevention of AHPND spread. Several one-step PCR methods target either the *Pir*^*vp*^*A* gene or *Pir*^*vp*^*B* gene [5, 6, 8, 9], while the AP4 nested PCR method targets both the *Pir*^*vp*^*A* and *Pir*^*vp*^*B* genes [10]. The total assay detection time for these methods may require more than 8–12 h including steps of enrichment (for the 1-step method), DNA extraction, PCR amplification and amplicon detection by electrophoresis. In contrast, loop-mediated isothermal amplification (LAMP) achieves synthesis of large amounts of DNA in a shorter time and in a simpler manner without sacrificing sensitivity or specificity, and it requires only a heating block or hot water bath rather than an expensive thermocycler.

LAMP amplicons are usually detected by agarose gel electrophoresis (LAMP-AGE), followed by staining with carcinogenic ethidium bromide as described in a recent VP_AHPND_ detection method [11]. To speed up the process by avoiding electrophoresis and to confirm the LAMP amplicons by a hybridization step, detection can be achieved using DNA-functionalized gold nanoparticles (AuNP) [12–15]. AuNPs chemically functionalized with alkyl thiol-terminated oligonucleotides are highly stable in saline solutions and can hybridize with complementary nucleic acids in a very selective and cooperative manner [16]. AuNPs exhibit characteristics of a surface plasmon resonance (SPR) absorption band in the visible light region with the spectrum dependent upon the inter-particle distance. Specifically, particle aggregation gives rise to a shift of the SPR absorption band and a concomitant red to purple-blue color change. This property has been utilized for solution-phase colorimetric detection of specific nucleic acid sequences [12–15]. In this manner, the detection method not only makes the amplicons visible by the unaided eye but also has the advantage of confirming their identity by DNA hybridization.

In this paper, LAMP was combined with use of an ss-DNA-labeled AuNP probe for detection of a *Pri*^*vp*^*A* target gene sequence in DNA extracts from VP_AHPND_ bacteria or from shrimp infected with them. Visual detection of the LAMP amplicons by the unaided eye was based on their ability to hybridize with the complementary gold-bound ss-DNA and thus prevent the normal red to purple-blue color change that would otherwise occur by salt-induced aggregation of the gold particles, as shown in Fig 1. The LAMP method combined with amplicon detection by AuNP has advantages over previously published methods for VP_AHPND_ detection by PCR or LAMP followed by electrophoresis in terms of reduced assay time, amplicon confirmation by hybridization and use of simpler equipment (i.e., no need for a thermocycler, electrophoresis equipment or a UV trans-illuminator.

**Fig 1:** Schematic illustration of the detection of VP_AHPND_ using DNA-functionalized gold nanoparticles as colorimetric hybridization probes to detect complementary LAMP amplicons. (1) Positive reaction for VP_AHPND_. (2) Negative reaction for VP_AHPND_.

## Materials and Methods

### Bacterial strains and DNA preparation

A total of 89 bacterial isolates were used. These included 77 isolates of *V*. *parahaemolyticus* obtained from shrimp, shrimp pond water or shrimp pond sediments. After isolation, all were tested for ability to cause AHPND by the laboratory bioassay of Tran et. al. (2015) [3] and 50 isolates were found to cause AHPND (VP_AHPND_ isolates) while 27 isolates did not (non-AHPND bacterial isolates), as previously reported [5,17]. An additional set of 7 isolates representing other *Vibrio* species commonly found in diseased shrimp in Thailand and 6 isolates representing non-*Vibrio* species were obtained from culture collections. A summary of these isolates is given in Table 1. *Bacillus subtilis* was included because it is often used as a shrimp probiotic, and the other 4 isolates were included because of our unpublished results indicating their possible presence in shrimp from EMS ponds. The isolates were stored at -80°C and re-streaked on suitable agar plates as previously described [18,19]. In brief, all *Vibrio* isolates were cultured on thiosulfate citrate bile salt sucrose agar (TCBS agar; Difco) containing additional 1.5% NaCl, while non-*Vibrio* isolates were cultured on tryptic soy agar (TSA; Difco) and incubated at 37°C overnight. Although it is customary to cultivate *Vibrio* pathogens of shrimp at 28–30°C for pathology studies with shrimp, the objective of our cultivation was to obtain DNA extracts only, and all the isolates we used grew sufficiently well at 37°C for this purpose. We selected 37°C for convenience related to limitations in incubator space. Bacterial DNA was extracted from a single loop of cells from these agar cultures using a Genomic DNA Purification Kit (Fermentas) according to the manufacturer’s protocol. The concentration and quality of the extracted DNA were analyzed by spectrophotometer at 260 and 280 nm and kept at -80°C until used.

**Table 1:** Bacterial isolates used in this study.

Bacterial isolates	Bioassaytest	Amplification			Origin	Source
		NestedPCR	LAMP-AGE	LAMP-AuNP		
*V*.*parahaemolyticus*						
1D	✓	**+**	**+**	**+**	*P*. *vannamei*	Centex
3HP	✓	**+**	**+**	**+**	*P*. *vannamei*	Centex
5HP	✓	**+**	**+**	**+**	*P*. *vannamei*	Centex
SA	✗	**−**	**−**	**−**	Shrimp pond	DMST
SB	✗	**−**	**−**	**−**	Shrimp pond	DMST
CHN	✓	**+**	**+**	**+**	*P*. *vannamei*	Centex
F1-CP	✓	**+**	**+**	**+**	*P*. *vannamei*	CP
F2-CP	✓	**+**	**+**	**+**	*P*. *vannamei*	CP
F3-CP	✓	**+**	**+**	**+**	*P*. *vannamei*	CP
F4-CP	✓	**+**	**+**	**+**	*P*. *vannamei*	CP
F5-CP	✓	**+**	**+**	**+**	*P*. *vannamei*	CP
F6-CP	✓	**+**	**+**	**+**	*P*. *vannamei*	CP
F7-CP	✓	**+**	**+**	**+**	*P*. *vannamei*	CP
F8-CP	✓	**+**	**+**	**+**	*P*. *vannamei*	CP
F9-CP	✓	**+**	**+**	**+**	*P*. *vannamei*	CP
F10-CP	✓	**+**	**+**	**+**	*P*. *vannamei*	CP
F11-CP	✗	**−**	**−**	**−**	*P*. *vannamei*	CP
F12-CP	✗	**−**	**−**	**−**	*P*. *vannamei*	CP
F13-CP	✗	**−**	**−**	**−**	*P*. *vannamei*	CP
F14-CP	✗	**−**	**−**	**−**	*P*. *vannamei*	CP
F15-CP	✗	**−**	**−**	**−**	*P*. *vannamei*	CP
F16-CP	✗	**−**	**−**	**−**	*P*. *vannamei*	CP
F17-CP	✗	**−**	**−**	**−**	*P*. *vannamei*	CP
F18-CP	✗	**−**	**−**	**−**	*P*. *vannamei*	CP
F19-CP	✗	**−**	**−**	**−**	*P*. *vannamei*	CP
F20-CP	✓	**+**	**+**	**+**	*P*. *vannamei*	CP
F21-CP	✗	**−**	**−**	**−**	*P*. *vannamei*	CP
VP1-CP	✗	**−**	**−**	**−**	*P*. *vannamei*	CP
VP2-CP	✗	**−**	**−**	**−**	*P*. *vannamei*	CP
VP3-CP	✓	**+**	**+**	**+**	*P*. *vannamei*	CP
VP4-CP	✓	**+**	**+**	**+**	*P*. *vannamei*	CP
VP5-CP	✗	**−**	**−**	**−**	*P*. *vannamei*	CP
VP6-CP	✓	**+**	**+**	**+**	*P*. *vannamei*	CP
VP7-CP	✓	**+**	**+**	**+**	*P*. *vannamei*	CP
VP8-CP	✓	**+**	**+**	**+**	*P*. *vannamei*	CP
VP9-CP	✓	**+**	**+**	**+**	*P*. *vannamei*	CP
VP10-CP	✗	**−**	**−**	**−**	*P*. *vannamei*	CP
UN1-CP	✗	**−**	**−**	**−**	*P*. *vannamei*	CP
UN2-CP	✗	**−**	**−**	**−**	*P*. *vannamei*	CP
UN3-CP	✓	**+**	**+**	**+**	*P*. *vannamei*	CP
UN4-CP	✓	**+**	**+**	**+**	*P*. *vannamei*	CP
UN5-CP	✗	**−**	**−**	**−**	*P*. *vannamei*	CP
UN6-CP	✓	**+**	**+**	**+**	*P*. *vannamei*	CP
UN7-CP	✓	**+**	**+**	**+**	*P*. *vannamei*	CP
UN8-CP	✗	**−**	**−**	**−**	*P*. *vannamei*	CP
UN9-CP	✓	**+**	**+**	**+**	*P*. *vannamei*	CP
UN10-CP	✓	**+**	**+**	**+**	*P*. *vannamei*	CP
CAAHRI1-CP	✓	**+**	**+**	**+**	*P*. *vannamei*	CP
CAAHRI2-CP	✓	**+**	**+**	**+**	*P*. *vannamei*	CP
CAAHRI3-CP	✓	**+**	**+**	**+**	*P*. *vannamei*	CP
CAAHRI4-CP	✓	**+**	**+**	**+**	*P*. *vannamei*	CP
CAAHRI5-CP	✓	**+**	**+**	**+**	*P*. *vannamei*	CP
CAAHRI6-CP	✓	**+**	**+**	**+**	*P*. *vannamei*	CP
CAAHRI7-CP	✓	**+**	**+**	**+**	*P*. *vannamei*	CP
CAAHRI8-CP	✓	**+**	**+**	**+**	*P*. *vannamei*	CP
CAAHRI9-CP	✗	**−**	**−**	**−**	*P*. *vannamei*	CP
CAAHRI10-CP	✓	**+**	**+**	**+**	*P*. *vannamei*	CP
CAAHRI11-CP	✓	**+**	**+**	**+**	*P*. *vannamei*	CP
CAAHRI12-CP	✗	**−**	**−**	**−**	*P*. *vannamei*	CP
CAAHRI13-CP	✗	**−**	**−**	**−**	*P*. *vannamei*	CP
CAAHRI14-CP	✗	**−**	**−**	**−**	*P*. *vannamei*	CP
CAAHRI15-CP	✓	**+**	**+**	**+**	*P*. *vannamei*	CP
CAAHRI16-CP	✓	**+**	**+**	**+**	*P*. *vannamei*	CP
CAAHRI17-CP	✓	**+**	**+**	**+**	*P*. *vannamei*	CP
CAAHRI18-CP	✓	**+**	**+**	**+**	*P*. *vannamei*	CP
CAAHRI19-CP	✗	**−**	**−**	**−**	*P*. *vannamei*	CP
CAAHRI20-CP	✓	**+**	**+**	**+**	*P*. *vannamei*	CP
CAAHRI21-CP	✓	**+**	**+**	**+**	*P*. *vannamei*	CP
CAAHRI22-CP	✓	**+**	**+**	**+**	*P*. *vannamei*	CP
CAAHRI23-CP	✓	**+**	**+**	**+**	*P*. *vannamei*	CP
CAAHRI24-CP	✓	**+**	**+**	**+**	*P*. *vannamei*	CP
CAAHRI25-CP	✓	**+**	**+**	**+**	*P*. *vannamei*	CP
CAAHRI26-CP	✗	**−**	**−**	**−**	*P*. *vannamei*	CP
CAAHRI27-CP	✓	**+**	**+**	**+**	*P*. *vannamei*	CP
CAAHRI28-CP	✗	**−**	**−**	**−**	*P*. *vannamei*	CP
CAAHRI29-CP	✓	**+**	**+**	**+**	*P*. *vannamei*	CP
CAAHRI30-CP	✓	**+**	**+**	**+**	*P*. *vannamei*	CP
*V*. *vulnificus*						
VVS4907001	✗	**−**	**−**	**−**	*P*. *vannamei*	DBSWU
VVS4907011	✗	**−**	**−**	**−**	*P*. *vannamei*	DBSWU
*V*. *harveyi*						
Centex639	✗	**−**	**−**	**−**	*P*. *monodon*	Centex
Centex1526	✗	**−**	**−**	**−**	*P*. *monodon*	Centex
*V*. *alginolyticus*						
DMST22082	✗	**−**	**−**	**−**	Stool (human)	DMST
DMST22084	✗	**−**	**−**	**−**	Food (human)	DMST
DMSC14800	✗	**−**	**−**	**−**	Seafood (human)	DMSC
*B*. *subtilis*	✗	**−**	**−**	**−**	Shrimp probiotic	Centex
*Shewanella* sp.	✗	**−**	**−**	**−**	*P*. *vannamei*	Centex
*Rhodococcus fascians*	✗	**−**	**−**	**−**	Not specified	NCCB
*Delftia acidovorans*	✗	**−**	**−**	**−**	Soil	NCCB
*Ralstonia solanacearum*	✗	**−**	**−**	**−**	Soil	Kasetsart

Centex: CENTEX Shrimp, Faculty of Science, Mahidol University, Bangkok, Thailand

DMST: Department of Medical Science, Ministry of Public Health, Thailand

DBSWU: Department of Biology, Faculty of Science, Srinakharinwirot University, Thailand

DMSC: Department of Microbiology, Faculty of Science, Chulalongkorn University, Thailand

CP: Aquatic Animal Health Research Center, Charoen Pokphand Co. Ltd, Thailand

NCCB: The Netherlands Culture Collection of Bacteria, CBS, Delft, the Netherlands

Kasetsart: Dr. J. Watcharachaiyakup, Kasetsart University, Kamphaengsaen Campus, Thailand

✓, AHPND pathology; ✗, no AHPND pathology; +, Positive reaction; **−**, negative reaction.

### Preparation of AuNPs

The colloidal solution containing AuNPs with an average diameter of 15 nm ± 3.5 nm was prepared as previously reported with minor modifications [15,20]. In brief, all glassware was thoroughly cleaned in *aqua regia* cleaning solution (three parts HCl and one part HNO_3_), rinsed in double-distilled water and oven dried prior to use. In a 250 ml round-bottom flask, 100 ml of a 1 mM solution of HAuCl_4_ (Sigma-Aldrich, USA) in double-distilled water was brought to a boil with vigorous stirring followed by the addition of 10 ml of 40 mM trisodium citrate (Sigma-Aldrich, USA). The solution turned deep blue immediately but later changed to a final wine-red. After this color change, boiling was continued for an additional 15 min before the heater was turned off and the colloidal AuNP solution was continuously stirred overnight. The resulting solution of AuNPs was characterized by an absorption maximum at 520 nm and it was stored in dark bottles at 4°C.

### Preparation of DNA-labelled AuNP probes

An ssDNA probe sequence was designed to complement that which spanned the F1c-B1c region of the AHPND-LAMP amplicon. It was labelled with a thiol group at the 5’-end (Table 2). The DNA-labelled AuNPs were prepared as previously described [12–15] with slight modifications. In brief, 10 ml of the colloidal AuNP solution was incubated with 5 nmol (i.e., 50 μl of the 100 μM stock) of 5’-thiol-modified ssDNA probes at 50°C with shaking at 150 rpm for 22 h. Then, the solution was transferred to 1 ml of phosphate buffer (100 mM sodium phosphate buffer, PH 7.6) containing 1 M NaCl and 10% SDS and incubated under the same conditions for another 4 h. The AuNPs were pelleted by centrifugation at 20,000 g at 4°C for 30 min to remove the unbound ssDNA. The supernatant solution was removed and the pelleted DNA-labelled AuNPs were washed with 5 ml washing buffer (100 mM PBS, 100 mM NaCl, 0.01% SDS) and finally re-suspended in 1 ml of the same buffer and kept at 4°C until used.

**Table 2:** Primers and probe used for LAMP to detect VP_AHPND_.

Primer name	Sequence (5’-3’)	Length (bp)
F3-EMS	GTGCAATTTAATAGGAGAACATC	23
B3-EMS	GAATGGTAAGCTCCCCAC	18
FIP-EMS	CGTTTGGTTCGACAGTCCAATTTTTATGAGTAACAATATAAAACATGA	48
BIP-EMS	GAGGCGTCACAGAAGTAGACATTTTCCCGTATTCTCAATGTCTACAC	47
LF-EMS	CGTGAGAATAGTCAGTT	17
LB-EMS	ACATACACCTATCATCCCGGAAG	23
Probe-Thiol-EMS	(SH)A_10_-ATCATCCCGGAAGTCGGTCG	30

### LAMP primer design and optimization

A set of six primers was designed for LAMP to target eight distinct regions of the *Pir*^*vp*^*A* gene of VP_AHPND_ isolates according to the sequence of GenBank accession no. KM067908.1 using Primer Explorer ver. 4 (http://primerexplorer.jp/lamp4.0.0/index.html). The sequences of the primers and their locations are indicated in Table 2. All primers were synthesized by Bio Basic Inc., Canada. To determine the optimal temperature for the LAMP assay, reactions were performed on a thermal cycler (Gene Amp PCR System 2700, Applied Biosystems^™^) at 60, 63 and 65°C for 1 h, followed by 85°C for 7 min to terminate the reaction. The products were analyzed by 2% agarose gel electrophoresis (AGE). The LAMP reaction mixtures (25 μl) consisted of 0.2 μM outer primers (F3 and B3), 2 μM inner primers (FIP and BIP), 0.2 μM loop primers (LF and LB), 0.4 M betaine (USB Corporation, USA), 1.2 mM dNTPs (Promega, USA), 6 mM MgSO_4_ (Sigma-Aldrich, USA), 8 U *Bst* DNA polymerase large fragment with the 1x buffer supplied (New England Biolabs, USA) and the specified amount of template DNA. DNA extracted from uninfected shrimp samples and sterile water were included as negative controls, and DNA extracted from the VP_AHPND_ isolate 5HP [17] was used as a positive control. To test specificity of the LAMP primers, DNA templates from 80 bacterial cultures (Table 1) were used to test the LAMP assay followed by both AGE and AuNP probe analysis.

### Optimization of the AuNP-probe hybridization step

The conditions for optimization of AuNP-probe hybridization were previously described [12–15] Briefly, hybridization for the detection of LAMP products was conducted in a total volume of 15 μl by mixing together the AuNP probe solution (5 nM) with the LAMP product solution at various ratios ranging from [1 μl AuNP solution: 9 μl product solution (1:9)] to [9 μl AuNP solution: 1μl product solution (9:1)] before incubation at 65°C for 5 min. After determining the optimum ratio, the conditions for salt-induced AuNP probe aggregation were determined using salt concentrations ranging from 3 to 666 mM MgSO_4_ in a fixed volume of 5 μl. Results were compared using LAMP amplicons obtained using DNA templates extracted from AHPND-bacterial culture isolate 5HP (positive control) and using distilled water and DNA extracted from shrimp infected with white spot syndrome virus (WSSV) (non-complementary target DNA) as negative controls. Color changes (red to blue color) were compared by the unaided eye and by UV-visible spectrum analysis (Thermo Fisher Scientific).

### Detection of VP_AHPND_ by 1-step and nested PCR

The DNA extracted from bacterial samples was used as a template for PCR amplification by both 1-step and nested PCR detection methods targeting the *Pir*^*vp*^*A* gene. Conditions for the AP3 1-step PCR method were similar to those described in a previous report [5] with some modifications. The 336-bp target fragment was amplified with primers F-AP3 and R-AP3 (Table 3) using the cycling protocol of 94°C for 5 min followed by 30 cycles of 94°C for 30 s, 53°C for 20 s and 72°C for 40 s and a final extension step at 72°C for 5 min.

**Table 3:** Primers used for 1-step PCR (AP3 method) and nested PCR (AP4 method) for detection of VP_AHPND_.

Primer name	Sequence (5’-3’)	Length (bp)
F-AP3	ATGAGTAACAATATAAAACATGAAAC	26
R-AP3	GTGGTAATAGATTGTACAGAA	21
F1-AP4	ATGAGTAACAATATAAAACATGAAAC	26
R1-AP4	ACGATTTCGACGTTCCCCAA	20
F2-AP4	TTGAGAATACGGGACGTGGG	20
R2-AP4	GTTAGTCATGTGAGCACCTTC	21

The two-tube nested PCR method (AP4) was carried out as in a previous report [10] with some modifications. The first-step PCR target of 1269-bp was amplified using primers AP4-F1 and AP4-R1 (Table 3), and this amplicon was then used as the template for a second PCR reaction that yielded a 230-bp amplicon using primers AP4-F2 and AP4-R2 (Table 3). Each PCR reaction was conducted in a 25 μl reaction mixture containing 1 x PCR buffer, 0.2 mM dNTPs (Promega), 3 mM MgCl_2_ (Invitrogen), 1.5 units *Taq* DNA polymerase (Invitrogen), 0.2 μM each forward and reverse primer, and 2 μl of template DNA. The PCR amplification was conducted with an initial cycle at 94°C for 2 min followed by 30 cycles of 94°C for 20 s, 55°C for 30 s and 72°C for 90 s (for external primers) or 20 s (for internal primers) followed by an extension step at 72°C for 2 min.

### Comparison of sensitivity between LAMP-AuNP and traditional PCR assays

The sensitivity comparison was carried out using tenfold serial dilutions of DNA extracted from pure cultures of VP_AHPND_ isolate 5HP at concentrations ranging from 10^7^ to 1 CFU/ml and prepared as previously described [18,19] with some modifications. Briefly, a small number of cells from a single bacterial colony on TCBS agar was inoculated into 5 ml of tryptic soy broth (TSB; Difco) supplemented with 1.5% NaCl and incubated overnight at 37°C. Then, 50 μl of this TSB culture was transferred into a new tube containing 5 ml of TSB followed by incubation at 37°C with shaking at 250 rev min^-1^ to obtain mid-log phase cells (OD_600 nm_ = 0.5). Tenfold serial dilutions of these cultures were prepared in phosphate buffered saline solution (PBS).

DNA template was prepared from these dilutions by transferring 100 μl from each dilution into a 1.5 ml microcentrifuge tube that was centrifuged at 15,000 g for 5 min. After removal of the supernatant, the pellets were subjected to DNA extraction using a Genomic DNA Purification Kit (Fermentas) according to manufacturer’s protocol. The resulting DNA extracts were used as templates for the LAMP-AuNP method and for the AP3 and AP4 PCR methods. The sensitivity tests were carried out in triplicate, and the last dilution that gave positive results with all three of the replicates was considered to be the detection limit for each method.

In parallel with the above, 100 μl aliquots of each dilution were spread on TSA supplemented with 1.5% NaCl (in duplicate) and the plates were incubated overnight at 37°C to determine bacterial counts. After colonies were visible, plates for counting were selected from dilutions that yielded 30–300 colony-forming units (CFUs) and these counts were used to calculate the CFU ml^-1^ of all the bacterial suspensions used.

### Specificity of the LAMP-AuNP assay for VP_AHPND_ detection

To test for cross-hybridization using the AuNP probe with LAMP products from other pathogens, the amplicons from a VP_AHPND_ DNA template (this study) served as the positive control for analysis by the AuNP colorimetric assay (analyzed by naked eye and confirmed by UV-vis spectrophotometry). The results were compared with those obtained using LAMP or RT-LAMP amplicons obtained by comparable LAMP methods for the following non-shrimp pathogens *Mycobacterium tuberculosis* (TB) [21] and *Plasmodium* (Malaria) [22], and for the shrimp pathogens WSSV [23], YHV [12], IMNV [13], IHHNV [24], TSV [25], LSNV [26] and PemoNPV [27].

### Evaluation of the LAMP-AuNP method for VP_AHPND_ detection in field samples

It has previously been recommended that shrimp and environmental samples to be tested for VP_AHPND_ using the AP3, 1-step PCR method should be subjected to a preliminary culture enrichment step to avoid false negative test results [5]. The subsequent AP4, nested PCR detection method was developed for testing samples that could not be enriched before testing (e.g., samples preserved in alcohol or archived DNA samples) [10]. Thus, we wished to compare the test results of these two methods with the LAMP-AuNP method to determine whether it might be used for the same purpose as the AP4 method for DNA extracts derived directly from shrimp stomach tissue (i.e., no enrichment step). Samples including 20 black tiger shrimp and 10 whiteleg shrimp were arbitrarily selected from shrimp farms where some VP_AHPND_ specimens had been previously detected. They were kindly provided by the Charoen Pokphand Foods (CPF) PCL Laboratory. The samples themselves were of unknown VP_AHPND_ infection status. Stomach tissue from individual shrimp was used for DNA extraction as described above. The extracted DNA was then used as the template for VP_AHPND_ detection by the LAMP-AuNP method and by the AP3 1-step and AP4 nested PCR methods. Then, the results for each method were compared.

## Results and Discussion

### Optimization of the reaction for VP_AHPND_ detection by LAMP

Tests for the optimal LAMP reaction temperature using 100 ng of DNA template from the VP_AHPND_ isolated 5HP revealed that 65°C gave a slightly better result by AGE analysis than 60 or 63°C (Fig 2). Thus, 65°C was selected as the standard assay temperature. When the LAMP reactions were conducted at 65°C for 30, 45 and 60 min using various concentrations of DNA template, the 45 and 60 min reaction times gave clear LAMP amplicon patterns of the same intensity while 30 min yielded pattern of lower intensity (data not shown). Thus, the shortest reliable time of 45 min was chosen as the standard assay time.

**Fig 2:** Optimization of the LAMP assay for detection of VP_AHPND_ at different temperatures (60, 63 and 65°C) using 100 ng of DNA extracted from VP_AHPND_ isolate 5HP in duplicate tests (Lane P). Lane M: 2 log DNA marker, Lane N: 100 ng of DNA extracted from healthy *P*. *monodon* (negative control).

### AuNP synthesis and hybridization for detection of VP_AHPND_ LAMP amplicons

Successfully synthesized AuNPs gave a UV-Vis spectrum with one peak at 525 nm (Fig 3), while the ssDNA-labelled AuNPs absorbed at 530 nm (Fig 3). This wavelength shift confirmed that the preparation contained monodispersed AuNPs.

**Fig 3:** Comparison of absorption spectra of colloidal AuNP and of the DNA-labelled AuNP probe.

Tests of the effect on hybridization when using a 5 nM AuNP solution at variable ratios with a LAMP product solution revealed that the best hybridization and aggregation result after addition of 50 mM MgSO_4_ was obtained using a mixture of the AuNP probe solution and LAMP product solution at a ratio of 5:5. This gave the clearest color difference between the positive red result and negative purple-blue result (Fig 4A).

**Fig 4:** Optimization of AuNP hybridization for detection of VP_AHPND_ amplicons. (A) Effect of variation in the volume ratio of the AuNP probe solution (5 nM) and the VP_AHPND_ LAMP amplicon solution from 1:9 to 9:1 (gold probe:Lamp amplicon) followed by addition of 50 mM MgSO_4_ and showing that 5:5 was the best ratio. (B) Effect of variation in MgSO_4_ concentration (between 3 and 667 mM in a fixed volume) in tubes with a gold probe: Lamp amplicon ratio of 5:5 and containing either (1) VP_AHPND_ LAMP amplicon or (2) WSSV LAMP amplicon (non-complementary DNA target negative control) or (3) LAMP premix without DNA target (no-target negative control) and showing that 50 mM gave the best result.

After optimizing the ratio of the AuNP probe and LAMP product solutions, tests needed to optimize the MgSO_4_ concentration to obtain the best visible test result from AuNP aggregation revealed that a final concentration of 50 mM was the most suitable (Fig 4B). It gave a distinct red positive result for VP_AHPND_-LAMP amplicons and a clearly contrasted purple-blue negative result for the distilled water and non-target DNA probe negative controls. Lower concentrations of MgSO_4_ (3 to 17 mM MgSO_4_) resulted in false-positive results (pink color) with the negative controls, while higher concentrations (100 and 667 mM MgSO_4_) resulted in false negative results (purple-blue/clear) with LAMP amplicons from VP_AHPND_ (Fig 4B). Therefore, the optimal MgSO_4_ concentration chosen in this study was 50 mM.

### Comparative sensitivity of LAMP-AuNP and PCR-electrophoresis methods

Using DNA extracts from ten-fold serial dilutions of VP_AHPND_ isolate 5HP, the LAMP-AuNP method was able to detect 5HP in a solution containing 100 CFU/ml (Fig 5A). This result showed similar sensitivity to LAMP-AuNP followed by UV-Vis analysis (Fig 5B), LAMP followed by AGE (Fig 5C) and nested-PCR using the AP4 method that amplifies a 230-bp fragment (Fig 6A). By contrast, the AP3, 1-step PCR method required a solution containing 10^4^ CFU/ml to obtain a positive result (Fig 6B). Another advantage of the LAMP-AuNP method was the short, total assay time of 50 min (45 min for LAMP, 5 min for hybridization and less than 1 min salt-induced aggregation). This compared to 90–120 min for the LAMP-AGE method, 3–5 h for the AP3, 1-step PCR method (excluding enrichment that might be required for natural samples) and 4–6 h for the AP4 nested-PCR method.

**Fig 5:** Sensitivity of the LAMP-AuNP assay for the detection of VP_AHPND_ using 10-fold serial dilution of DNA extracted from a culture of VP_AHPND_ isolate 5HP (10^7^−1 CFU/ml). (A) Colorimetric results of LAMP followed by AuNP probe assay. (B) UV-visible spectrum analysis corresponding to the individual tubes in Fig 5A (measured after salt addition). (C) AGE results of LAMP reactions. Lane M: 2 log DNA marker and N: 100 ng of DNA extracted from normal shrimp.

**Fig 6:** Comparison of a sensitivity test carried out using total DNA template as in Fig 5 with traditional PCR methods. (A) Nested PCR followed by AGE (AP4 method). (B) 1-step PCR followed by AGE (AP3 method). Lane M: 2 log DNA marker and N: 100 ng of DNA extracted from normal shrimp.

### Specificity of LAMP-AuNP for VP_AHPND_ detection

Tests for cross hybridization using the AuNP probe with amplicons produced using LAMP methods for other shrimp pathogens (Fig 7A) gave no positive results using the AHPND AuNP probe (Fig 7B). Instead, the LAMP-AuNP assay gave a red positive result only with the LAMP product from the VP_AHPND_ isolate. The color of the positive LAMP-AuNP test result was stable over 30 min after salt addition, while LAMP products from other pathogens gave an immediate color change to purple-blue followed by precipitation of the aggregated probe to yield a colorless supernatant solution within 30 min (not shown). The results by UV-Vis detection for the red nanogold probe showed identical specificity results (Fig 7C) to those using the unaided eye (Fig 7B).

**Fig 7:** Comparison of results obtained using the VP_AHPND_ AuNP hybridization probe with LAMP amplicons from VP_AHPND_ (Lane 1) and other common pathogens (Lanes 2–10). (A) The result of agarose gel electrophoresis (AGE) of LAMP products from various pathogens. Lane M: 2 log DNA marker; Lane N: normal shrimp DNA as negative control; Lanes 2–10: TB, *Plasmodium* (Malaria), WSSV, YHV, IMNV, IHHNV, TSV, LSNV and PemoNPV, respectively. (B) Colorimetric result for the same LAMP products as in Fig 7A measured after salt addition. (C) UV-visible spectra analysis corresponding to the individual tubes in Fig 7B measured after salt addition.

### Detection of VP_AHPND_ using LAMP-AuNP, LAMP-AGE and nested PCR with DNA from pure cultures of various bacterial isolates

Testing the specificity of LAMP-AuNP for detection of VP_AHPND_ with DNA templates from 89 bacterial isolates (Table 1) revealed that both the LAMP-AuNP assay and nested PCR assay gave positive test results for all 50 VP_AHPND_ isolates but negative results for the 40 non-AHPND isolates. The LAMP-AGE assay also gave positive test results for all the VP_AHPND_ isolates and negative results for all the non-AHPND isolates.

### Comparison of LAMP-AuNP and PCR methods for detection of VP_AHPND_ in field samples

These tests were carried out using 30 samples of shrimp of unknown VP_AHPND_ infection status arbitrarily selected from shrimp farms were shrimp infected with VP_AHPND_ had been detected previously. The purpose was to test whether the LAMP-AuNP method could be used similarly to the AP4 PCR method to detect VP_AHPND_ in shrimp or other specimens without the culture enrichment step usually employed prior to using the AP3, 1-step PCR detection method. Using direct DNA extracts from the stomachs of the shrimp specimens as templates, 7 of the 30 shrimp (2 black tiger shrimp and 5 whiteleg shrimp) (23.3%) gave positive test results for VP_AHPND_ using the 1-step PCR AP3 method. In contrast, 12 of the 30 samples (7 more for a total 40%) gave positive test results for VP_AHPND_ by both the LAMP-AuNP and the AP4 nested-PCR methods (Table 4). Together with the results on comparative sensitivity described in the preceding section above, these results showed that the LAMP-AuNP method has similar utility to the AP4 nested PCR method in detecting VP_AHPND_ in samples where the target DNA is too low in concentration to be detected directly by a representative 1-step PCR method. This test was not carried out to determine the prevalence of such lightly-infected samples that might occur in field testing for VP_AHPND_, but to show that the LAMP-AuNP method can be used to test samples that are not enriched before testing. At the same time, it is clear that the LAMP-AuNP was faster and simpler to use in farm-site laboratories than the AP4 method.

**Table 4:** Comparison of detection results for VP_AHPND_ in field samples using LAMP combined with AuNP, 1-step PCR (AP3 method) and nested PCR (AP4 method).

		Number (%) of positive results		
Type of sample	No. of samples	1-PCR	Nested PCR	LAMP-AuNP
Whiteleg shrimp	10	2 (20.0)	4 (40.0)	4 (40.0)
Black tiger shrimp	20	5 (25.0)	8 (40.0)	8 (40.0)
Total	30	7 (23.3)	12 (40.0)	12 (40.0)

### Overall conclusions for the LAMP-AuNP method to detect VP_AHPND_

The initial detection methods for VP_AHPND_ were based on standard 1-step PCR detection of the pAP1 plasmid, but these methods gave a small percentage (~3%) of false positive results, probably due to absence of the Pir^vp^A and Pir^vp^B toxin genes on pAP1 plasmids of the bacteria being tested [5]. Subsequent 1-step PCR detection methods targeted either the Pir^vp^A or Pir^vp^B toxin [5, 6, 8,9] and none of those reports included any false negative or false positive results for VP_AHPND_ in the form of specimens that have tested positive or negative, respectively, for the Pir^vp^A or Pir^vp^B genes. In other words, all AHPND specimens positive for one of the toxins have also been positive for the other. This suggests that prevalence of the theoretically possible mutant specimens carrying only one or the other of the two toxin genes is very low and that for practical purposes only one of the toxin genes is sufficient for detection of VP_AHPND_. Indeed, the AP4 nested PCR method that targets both toxins has given identical results to those obtained using the AP3 1-step PCR method with large numbers of samples, and the two methods differ only in higher sensitivity of the nested PCR method [10].

More recently, a LAMP-AGE method for detection of VP_AHPND_ has been published [11], but compared to the LAMP-AuNP method, it has the disadvantages of requiring the use of electrophoresis equipment and lacking a hybridization step to confirm the specific nature of the LAMP amplicons. There are two other LAMP amplicon detection protocols (not yet reported for use in VP_AHPND_ detection) that do not use electrophoresis but give color reactions visible to the naked eye, like the LAMP-AuNP method. However, both lack a hybridization step to confirm the nature of the amplicons. These are the calcein method [28] and the hydroxynaphthol blue method [29], both of which measure accumulation of the phosphate byproduct of the LAMP reaction and could give false-positive color reactions with non-specific LAMP amplicons [30]. Similarly, the LAMP amplicon detection methods that involve use of the fluorescent, DNA-intercalating dye SYBR Green I, would also give positive fluorescence signals with non-specific amplicons, and they have the added requirement for a fluorescence spectrophotometer [31]. Thus, high sensitivity, high specificity including amplicon confirmation by hybridization, relatively short analysis time and use of simple equipment (i.e., no thermocycler, no electrophoresis equipment and no spectrophotometer) are the key advantages of the LAMP-AuNP detection method for VP_AHPND_. It is a rapid and relatively simple assay with sensitivity comparable to that of traditional nested-PCR detection but suitable for confirmation of AHPND outbreaks in small, farm-scale laboratories.
